# Inhibition of microRNA-218 reduces HIF-1α by targeting on Robo1 in mice aortic endothelial cells under intermittent hypoxia

This article has been retracted.

**DOI:** 10.18632/oncotarget.22239

**Published:** 2017-10-26

**Authors:** Kai-Xiong Liu, Qin Chen, Gong-Ping Chen, Jian-Chai Huang, Jie-Feng Huang, Xin-Ru He, Ting Lin, Qi-Chang Lin

**Affiliations:** ^1^ Department of Respiratory Disease, The First Affiliated Hospital, Fujian Medical University, China; ^2^ Laboratory of Respiratory Disease of Fujian Medical University, Fuzhou, China; ^3^ Fujian Provincial Sleep-disordered Breathing Clinic Center, Fuzhou, China; ^4^ Integrated Chinese and Western Medicine Colleges, Fujian University of Traditional Chinese Medicine, Fuzhou, China

**Keywords:** microRNA-218, intermittent hypoxia-inducible factor-1α, apoptosis, normal mice aortic endothelial cells

## Abstract

**Objective:**

To investigate the effects of miR-218 on expression of hypoxia-inducible factors 1α (HIF-1α), vascular endothelial growth factor (VEGF) and cell apoptosis in normal mice aortic endothelial cells under intermittent hypoxia (IH) condition.

**Methods:**

Anti-miR-218 inhibitor, miR-negative control and miR-218 mimic were used to tranfect the cells in different groups under IH condition. Both RT-PCR and Western blot were used to determine the expressions of HIF-1α and VEGF. Akt, p-Akt and cell apoptosis related proteins bcl-2, bax and caspase-3 and roundabout 1 (Robo1) were measured using Western blot. Cell apoptosis was evaluated by flow cytometry. Statistical analysis was performed using SPSS 18.0.

**Results:**

Expression of miR-218 was significantly up-regulated in the IH group and was significantly inhibited when cells were transfected with miR-218 inhibitor. Down regulation of miR-218 could reduce the expression of HIF-1α and VEGF under intermittent hypoxia condition. In cells transfected with miR-218 mimic, expression of HIF-1α and VEGF significantly increased compared with the control. However, when treated with LY294002, the expression of HIF-1α and VEGF both decreased. Apoptosis assay showed that down regulation of miR-218 could inhibit intermittent hypoxia induced cell apoptosis, decrease expression of caspase-3 and bax and increase expression of bcl-2 under intermittent hypoxia condition. At last, silencing Robo1 could significantly enhance the expression of HIF-1α under IH condition.

**Conclusion:**

Inhibition of miR-218 could reduce the expression of HIF-1α and protect against IH-induced apoptosis in mice aortic endothelial cells. The effects were associated with PI3K/AKT pathway and might through targeting of Robo1.

## INTRODUCTION

Obstructive Sleep Apnea (OSA), of which the main symptom is the repeated episodes of upper airway obstruction during sleep, is recognized as a significant and highly prevalent health problem with cardiovascular and metabolic morbidity, as well as its prominent cognitive and behavioral implications [1]. Studies have demonstrated that intermittent hypoxia (IH) is the key pathophysiological character of OSA [2, 3]. IH is associated with lots of biological process, including neurobehavioral impairments, increased apoptosis and oxidant stress and inflammation [4]. And cell apoptosis induced by IH is one of the main problems in OSA patients [4, 5].

Several studies suggested that IH influenced a variety of transcription factors, including the hypoxia-inducible factors 1α (HIF-1α), nuclear factor of activated T cells, activator protein 1 and NF-kB [6]. Recent studies have shown that HIF-1α is one of the major molecular mechanisms which increases ROS generation, regulates the expression of downstream target genes and mediates cell apoptosis caused by IH-induced endothelial injury [7]. What’s more, scientists found that IH could not only up-regulate the level of HIF-1α, but also the expression of vascular endothelial growth factor (VEGF) [8, 9].

MicroRNAs (miRNAs) are small endogenous RNAs involved in various biological process and diseases such as tumorigenesis, cell proliferation, apoptosis, and autophagy [10, 11]. Recent studies turned their eyes on the role of miRNAs in IH and found that several miRNAs could influence IH process and protected cells against hypoxia-induced apoptosis [12]. MiR-218 is a vertebrate-specific intronic miRNA which attracted lots of attentions in recent years. Studies show that miR-218 is frequently down-regulated in various cancers and acts as a tumor suppressor by targeting different proteins [13-15]. However, the role of miR-218 in IH has not been reported yet.

Our previous study has identified that OSA can up-regulate the concentration of HIF-1α in plasma, leading to the high-expression of VEGF and increase vascular density to adopt anoxia [16]. Besides, we used miRNA chip analysis and found that miR-218 was up-regulated during intermittent hypoxia in the previous study. In this study, we demonstrated that down-expression of miR-218 could reduce the expression of HIF-1α, VEGF and protect against intermittent hypoxia-induced apoptosis in normal mice aortic endothelial cells for the first time. Our data may be useful for further relative researches and contribute to development of a new therapy for OSA-associated endothelial dysfunction.

## RESULTS

### Down regulation of miR-218 significantly reduced expression of HIF-1α and VEGF under intermittent hypoxia

First, cells were divided into 4 groups: cells transfected with anti-miR-218 inhibitor and incubated under intermittent hypoxia; the negative group, cells transfected with miR-negative control and incubated under intermittent hypoxia; the IH group, cells incubated under intermittent hypoxia; and the normoxia cells, cells cultured under normoxia. Expression of miR-218 was determined using RT-PCR in different cell groups. Results showed that when treated under intermittent hypoxia condition, miR-218 was significantly increased compared to the normoxia cells, P<0.001. And when treated with miR-218 inhibitor, the interference significantly reduced its expression compared with the IH group, P<0.001, which showed successfully down regulation of miR-218 under IH (Figure 1). Then expressions of HIF-1α and VEGF were determined by both RT-PCR and Western blotting. Results showed that IH condition could significantly enhance the expression of both HIF-1α and VEGF compared with the normoxia cells, P<0.001, while down regulation of miR-218 significantly inhibited the increase of the two factors, P<0.001, indicating the regulating influence of miR-218 on HIF-1α and VEGF (Figure 2).

**Figure 1:** Expression of miR-218 in different cell groups. ^*^ P<0.05, compared with the IH group

**Figure 2:** **(A)** Expression of RNAs of HIF-1α and VEGF in different cell groups by RT-PCR. **(B and C)** Expression of HIF-1α and VEGF in different cell groups by Western blotting. ^*^ P<0.05, compared with the IH group.

### PI3K/Akt pathway was involved in regulation of miR-218 on expression of HIF-1α and VEGF

Studies showed that some other miRNAs, such as miR-494 and miR-21 could activate HIF-1α through PI3K/Akt pathway [12, 17]. In the present study, we used miR-218 mimic and PI3K inhibitor LY294002 to investigate the regulation mechanism of miR-218 on HIF-1α and VEGF. Cells in this section were divided into 4 different groups: the interference and negative groups, which were described above; the miR-218 mimic group, using miR-218 mimic to transfect cells; the miR-218 mimic and PI3K inhibitor group, which were transfected with miR-218 mimic and then treated with LY294002. Results showed that under IH condition, when treated with miR-218 mimic, the expression of HIF-1α and VEGF significantly increased compared with the negative control, P<0.001, which demonstrated that miR-218 could also increase the expression of the two factors (Figure 3A and 3B). Meanwhile, up regulating miR-218 could also enhance the expression of p-Akt (Figure 3B). However when LY294002 was added, the over expression effects of HIF-1α, VEGF and p-AKT induced by miR-218 were significantly inhibited compared with miR-128 mimic group, P<0.001. These results indicated that miR-218 may regulate the expression of HIF-1α and VEGF through PI3K/Akt pathway.

**Figure 3:** **(A)** Expression of RNAs of HIF-1α and VEGF in different groups. **(B and C)**. Expression of HIF-1α, VEGF and p-Akt in different cell groups by Western blotting. ^*^P<0.05, compared with the miR-218 mimic group.

### Down regulation of miR-218 reduced expression of caspase-3, bax and enhanced expression of bcl-2 under intermittent hypoxia

To investigate the influence of down regulation of miR-218 on cell apoptosis, expression of apoptosis related proteins bcl-2, bax and caspase-3 were evaluated using Western blotting. Results showed that when treated under IH condition, expression of caspase-3 and bax was significantly increased, P<0.001, while expression of bcl-2 was apparently decreased compared with the blank group, P<0.001, (Figure 4). However, when expression of miR-218 was interrupted, the above influence was significantly inhibited compared with the IH group, P<0.001,. These results suggested that down regulation of miR-218 could affect expression of cell apoptosis proteins.

**Figure 4:** **(A and B)** Expression of bcl-2, bax and caspase-3 in different cell groups by Western blotting. ^*^P<0.05, compared with the IH group.

### Down regulation of miR-218 inhibited intermittent hypoxia induced cell apoptosis

Then we determined cell apoptosis of different cell groups using flow cytometry. Results are shown in Figure 5. When treated with miR-218 inhibitor, cell apoptosis rate significantly decreased compared with the IH group, P<0.001,, in which the apoptosis rate significantly increased compared with the blank, P<0.001,. Combining with the alteration of apoptosis related proteins, we could deduce that down regulation of miR-218 could significantly inhibit the intermittent hypoxia-induced cell apoptosis.

**Figure 5:** **(A and B)** Cell apoptosis of different cell groups by flow cytometry. ^*^P<0.05, compared with the IH group.

### Robo1 was involved in the regulation of miR-218 on HIF-1α in mice aortic endothelial cells

Finally, we evaluated expression of Robo1 as possible target of miR-218. Several studies have reported that Robo1 was one of the targets of miR-218 (Figure 6A) [18], but few of them demonstrated relationship of Robo1 and miR-218 in endothelial cells. Here we confirmed that in normal endothelial cells, Robo1 was significantly down regulated when cells were transfected with miR-218 mimic and was significantly up regulated when cells were transfected with miR-218 inhibitor, P<0.05 (Figure 6B). In IH cells transfected with miR-218 inhibitor, expression of Robo1 was significantly higher than normal IH cells and expression of HIF-1α was significantly lower than normal IH cells. However, when IH cells were treated with both miR-218 inhibitor and si-Robo1, expression of HIF-1α significantly increased compared with the cells only treated with miR-218 inhibitor, P<0.001 (Figure 6C). These results indicated that miR-218 might regulate expression of HIF-1α targeting on Robo1.

**Figure 6:** **(A)** Conservation of the miR-218 binding site in Robo1, from ref [18]. **(B)**. Expression of Robo1 in different group of cells, ^*^P<0.05, compared with the NC group, ^#^P<0.05, compared with the miR-218 inhibitor group. **(C)**. Expression of HIF-1αin different group of cells, ^*^ P<0.05, compared with the miR-218 inhibitor group.

## DISCUSSION

It has been proved that intermittent hypoxia is the key pathophysiological character of Obstructive Sleep Apnea and the apoptosis that it induced is one of the main problems during the process. Relationships were found between the endothelial cells apoptosis in OSA patients and the endothelial dysfunction, but deeper mechanisms are still needed [19]. Studies showed that HIF-1α is one of the key factors involved in IH process. Evidences showed that continuous hypoxia could lead to accumulation of both HIF-1 and HIF-2 [20]. However, IH increases HIF-1 and decreases HIF-2 protein in cell cultures as well as in rodents [21]. Previous studies have shown that miR-218 could reduce HIF-2α through targeting multiple components such as EGFR, PLCγ1, PIK3C2A, and ARAF, but to our best knowledge, there are no studies focusing on relationship of miR-218 and intermittent hypoxia [22]. In this study, we tried to investigate the role of miR-218 in process of intermittent hypoxia and its effects on intermittent hypoxia induced apoptosis for the first time.

Results obtained in the present study are positive and encouraging. First we established a model of down regulated miR-218 in mice aortic endothelial cells under intermittent hypoxia condition and results showed the establishment was successful. In miR-218 interference group, expression of miR-218 was significantly reduced, while in intermittent hypoxia groups its expression increased significantly as expected.

Then we measured expression of HIF-1α and VEGF in different cell groups and the results clearly demonstrated the alteration of the two factors in different conditions. The IH condition could significantly enhance their expression and when miR-218 was interrupted the over expression was apparently inhibited. These results showed that miR-218 was closely related with expression of HIF-1α and VEGF. The up-regulated levels of HIF-1α and VEGF under IH condition were proved by lots of studies reported previously. Semenza et al reviewed role of HIF-1-dependent respiratory, cardiovascular, and redox responses to chronic intermittent hypoxia (CIH) and demonstrated that HIF-1 activity was induced when mice or cultured cells were subjected to CIH [23]. Briançon et al clearly showed that intermittent hypoxia could upregulate serum VEGF [24]. All these results are in consistent with the present study.

Then to further study the mechanism of the regulation effect of miR-218 on HIF-1α and VEGF, we used miR-218 mimic and PI3K inhibitor LY294002. Results showed that increased expression of miR-218 could also significantly induce the expression of HIF-1α and VEGF. Meanwhile, up-regulated miR-218 could enhance the expression of p-Akt, which can be inhibited by PI3K inhibitor, indicating that miR-218 might regulate the expression of HIF-1α and VEGF through PI3K/Akt pathway. Some similar studies have been reported before. Kanichai et al [25] studied a role for AKT and HIF-1αin rat mesenchymal stem cells under hypoxiacondition, results showed that hypoxia evoked an increase in phosphorylation of both AKT and p38 mitogen activated protein kinase, upstream of HIF-1α activation. Furthermore, the PI3 kinase/AKT inhibitor, LY294002 prevented the hypoxia-mediated stabilisation of HIF-1α. Martinive et al also demonstrated that under cyclic hypoxia condition, activation of the PI3K /Akt pathway during intervening reoxygenation periods was one of the major triggers of the stabilization of HIF-1α [26]. There are also studies which reported that miR-494 and miR-21 could also regulate HIF-1α through PI3K/Akt pathway [12, 17].

Studies showed that HIF-1α could induce the expression of downstream target genes, resulting in a series of hypoxic adaptation to achieve neuroprotection when mild hypoxia. But when cells were under chronic or severe hypoxia, HIF-1α would induce cell apoptosis [27]. In this study, the change of cell apoptosis was evaluated by both the flow cytometry and alteration of apoptosis related proteins. Over expression of HIF-1α was observed in cells under IH condition, as well as increased cell apoptosis. However, when miR-218 was down regulated, both of the above two effects were inhibited. Sun et al [12] demonstrated that over-expression of microRNA-494 could up-regulate HIF-1α and protects against hypoxia-induced apoptosis. But the influence of HIF-1α on apoptosis in intermittent hypoxia condition was rarely reported. In the present study, we demonstrated some possible relationships, though both continuous hypoxia and intermittent hypoxia can increase expression of HIF-1α, their influence on cell apoptosis may be different, however this hypothesis needs more studies to be further proved.

Finally, we evaluated expression of Robo1 as possible target of miR-218. Results showed that when IH cells were treated with both miR-218 inhibitor and si-Robo1, expression of HIF-1α significantly increased compared with the cells only treated with miR-218 inhibitor. These results indicated that to silence Robo1 could enhance the expression of HIF-1α, indicating that miR-218 might regulate expression of HIF-1α targeting on Robo1. Several studies have reported that Robo1 was one of the targets of miR-218 [18], but few of them demonstrated relationship of Robo1 and miR-218 in endothelial cells. Weigand et al demonstrated that Robo1 was decreased under hypoxia condition in endothelial cells [28]. All these results suggested that in endothelial cells miR-218 might also target on Robo1 under condition of hypoxia.

In conclusion, the present study determined the change of HIF-1α and VEGF when miR-218 was down regulated in mice aortic endothelial cells under intermittent hypoxia and studied the influence of down regulating miR-218 on intermittent hypoxia-induced cell apoptosis. Results showed that down-expression of miR-218 could significantly reduce the expression of HIF-1α and protect against intermittent hypoxia-induced apoptosis in mice aortic endothelial cells targeting on Robo1, which needs further investigation to get deeper insights.

## MATERIALS AND METHODS

### Cell culture and transfection

Mouse aortic endothelial cells were obtained as described previously [16]. Cells were maintained in RPMI 1640 medium (Gibco, Gaithersburg, MD, USA) supplemented with 10% fetal bovine serum (FBS). MiR-218 negative control, miR-218 mimic and inhibitor were all purchased from RiboBio, Guangzhou, China. Cells were grown under normoxic (21% O_2_) or hypoxic (1% O_2_) conditions at 37°C/5% CO_2_. To perform IH, cells were treated as described previously [16]. In the CIH group, cells were maintained at 37°C at 5% CO_2_ in a chamber (Oxycycler model A42, Biospherix) in which O_2_ levels were alternated between 21% for 5 min and 1% for 10 min, for a total of 64 cycles (18 h). Cells in the control group were maintained under normoxic condition. After hypoxic treatment, the medium was washed off, and the mouse aortic endothelial cells were returned to the maintenance medium (NCS-DMEM) in the normal incubator for 60-min recovery. Cells were cultured to 30-50% confluence and transfected with miR-218 inhibitor, negative control, miR-218 mimic or si-RNA and si-Negative Control (all purchased from RiboBio, Guangzhou, China) (10 nmol/L) using Lipofectamine 2000 (Invitrogen) in serum-free Opti-MEM medium (Gibco) according to the manufacturer’s instruction. Si-RNA of Robo1 was synthesed by Guangzhou Ribobio Co. Ltd. China. The sequence was: 5’-GAAAGCUCAUGAUCACUUAUAAGUGAUCAUGAGCUUUC-3’. PI3K inhibitor LY294002 was purchased from Sigma-aldrich, USA, and was added into the medium with concentration of 30 μmol/L to inhibit PI3K/Akt pathway. Transected cells were cultured for 48 hours under normoxia or IH.

### RNA extraction and real-time RT-PCR

The RNA extraction and reverse-transcription were performed as described elsewhere [29]. Briefly, Total RNA was extracted using TRIZOL reagent (Invitrogen, USA) according to the manufacturer’s instructions. A High Capacity cDNA Reverse Transcription Kit (Applied Biosystems, USA) was used to convert RNA into cDNA. Real-time PCR was conducted in an ABI7500 real-time PCR instrument (Applied Biosystems) with the SYBR Premix Ex Taq (TaKaRa). Primer sequences were as follows: HIF-1α forward 5’-CAAGAACCTACTGCTAATGC-3’, reverse 5’-TTATGTATGTGGGTAGGAGATG-3’; VEGF forward 5’-ACAGGGAAGAGGAGGAGATG-3’, reverse 5’-GCTGGGTTTGTCGGTGTTC-3’; GAPDH forward 5’-GAAGGTGAAGGTCGGAGTC-3’, reverse5’-GAAGATGGTGATGGGATTTC-3’.

### Western blot

Western blotting was used to test the expression of HIF-1α, VEGF and apoptosis related factors bcl-2, bax, caspase-3, and Robo1. GAPDH was used as a control. Samples extracted from the cells by normal method were loaded on SDS-PAGE and transferred to PVDF membranes. The membranes were then incubated with a primary antibody following with a conjugated secondary antibody. All antibodies used in the study were purchased from Abcam, Cambridge, UK. The films were scanned using Super Signal West Pico Chemiluminescent Substrate Kit (Pierce, Rockford, IL, USA) according to the manufacture’s instruction. The relative protein expression was analyzed by Image-Pro plus software 6.0.

### Flow cytometry

Cell apoptosis was analyzed using flow cytometry. Briefly, cells after IH were harvested and resuspended in culture media at a concentration of 1×10^6^ cells/mL. 300 μL of cell suspension were transferred to each centrifugal tube, 10μL of 30× FLICA working solution were added. Cells were then mixed and incubated for 60 minutes at 37°C, 5% CO_2_, washed and then centrifugated for 5 minutes. Then cells were resuspended in 400μL of 1×wash buffer, and stained with PI. Cell suspension was incubated for 5 minutes on ice in the dark. 400μL of stained cells were transferred to flow tubes and analyzed on the flow cytometer.

### Statistical analysis

All experiments were conducted in triplicate. All data were calculated by mean ± SD (standard deviation) and compared using ANOVA. Independent continuous variables were compared using the *t*-test. When *P*-value was less than 0.05 it was considered to be statistically significant. All calculations were made using SPSS 18.0.

Jie-Feng Huang, Xin-Ru He, Ting Lin and Qi-Chang Lin.
